The article "TTC7B Is a Novel Prognostic-Related Biomarker in Glioma Correlating with Immune Infiltrates and Response to Oxidative Stress by Temozolomide" was retracted in 2023. Reasons: signs of a paper mill; suspected computer-generated content; unreliable results or conclusions; concerns about the data.

# *TTC7B* Is a Novel Prognostic-Related Biomarker in Glioma Correlating with Immune Infiltrates and Response to Oxidative Stress by Temozolomide

**DOI:** 10.1155/2022/7595230

**Published:** 2022-09-20

**Authors:** Zhenhua Chen, Shasha Cui, Yong Dai, Chunfeng Lu, Huan Zhang, Wei Zhao, Hongyan Yan, Yi Zhang

**Affiliations:** ^1^Department of Neurosurgery, Affiliated Hospital 2 of Nantong University and First People's Hospital of Nantong City, North Haierxiang Road 6#, Nantong 226001, China; ^2^Nantong Health College of Jiangsu Province, East Zhenxing Road 288#, Nantong 226010, China

## Abstract

**Background:**

Gliomas are one of the most prevalent malignant brain tumors. Hence, identifying biological markers for glioma is imperative. *TTC7B* (Tetratricopeptide Repeat Domain 7B) is a gene whose role in cancer in currently identified. To this end, we examined the *TTC7B* expression as well as its prognostic significance, biological roles, and immune system impacts in patients with glioma.

**Methods:**

We evaluated the function of *TTC7B* in GBM and LGG through the published CGGA (Chinese Glioma Genome Atlas) and TCGA (The Cancer Genome Atlas) databases. CIBERSORT and TIMER were used to analyze the link between *TTC7B* and immune cells, while R was used for statistical analysis. In addition, Transwell analysis, including migration and invasion assays, was performed to identify the relationship between *TTC7B* and temozolomide.

**Results:**

Low expression of *TTC7B* was observed in GBM and LGG. 1p/19q codeletion, *IDH* mutation, chemotherapy, and grade were found to have a significant correlation with *TTC7B*. Besides, low *TTC7B* expression was linked with low overall survival (OS) in both GBM and LGG. In the Cox analysis, *TTC7B* was found to independently function as a risk element for OS of patients with glioma. Furthermore, CIBERSORT analysis demonstrated a positive link between *TTC7B* and multiple immune cells, especially activated NK cells. Transwell analysis, including migration and invasion assays, revealed that temozolomide reduced the migration and invasion capacity of glioma cells and increased the expression of *TTC7B*.

**Conclusion:**

In all, *TTC7B* could serve as a promising prognostic indicator of LGG and GBM, and is closely associated with immune infiltration and response to oxidative stress by temozolomide.

## 1. Introduction

Gliomas are among the most prevalent primary brain tumors in adults, accounting for over 70% of malignant brain tumors [1]. They have been categorized into three types: astrocytomas, oligodendrogliomas, and ependymomas on the basis of their histological characteristics and specific. World Health Organization (WHO) grades I-IV, which reflect the degree of malignancy [2–4]. The study of molecular mechanisms has led to a deeper understanding of gliomas. The codeletions of the chromosome arms 19q and1p, along with the molecular characterization of the primary brain tumors like *IDH* were included in gliomas as per the 2016 report of the WHO [3].

The article "TTC7B Is a Novel Prognostic-Related Biomarker in Glioma Correlating with Immune Infiltrates and Response to Oxidative Stress by Temozolomide" was retracted in 2023. Reasons: signs of a paper mill; suspected computer-generated content; unreliable results or conclusions; concerns about the data.

Although the current standard interventions, such as surgery, chemotherapy, and radiation, have improved the prognosis of patients with glioma [5, 6], it is still dismal. The local recurrence of tumor is closely associated with tumor heterogeneity, and the immune microenvironment of malignant tumor is a major reason for the failure of the treatment of malignant glioma [7]. Hence, new treatments for glioma are critical [8]. The molecular processes controlling the metabolism of glioma are rapidly developing, and are evidenced by a series of recent technological developments [9]. It is important to urgently elucidate these molecular mechanisms to develop new therapies to avail diagnosis and treatment of glioma.

In cellular signaling, metabolism, and epigenetics, reactive oxygen species (ROS) are essential regulators. The altered metabolism of cancer cells is generally characterized by increased glycolysis and ROS levels [10]. Growth of tumors and inflammation can further increase ROS, shifting the redox balance towards oxidation. When ROS levels are low to moderate, they may act as signaling molecules, induce DNA mutations, and inactivate tumor suppressor genes. When ROS are present at high levels, they cause cellular damage and death, a principle that has been exploited in cancer treatments involving ionizing radiation (IR) and chemotherapy [11].

*TTC7B* (Tetratricopeptide Repeat Domain 7B) is a protein-coding gene, which is linked to several diseases, including hypomyelinating leukoencephalopathy and trichohepatoenteric syndrome 1 [12]. Nonetheless, *TTC7B* has not been reported in patients with glioma to date. Moreover, the relation of *TTC7B* with the immune cell infiltration status in LGG and GBM is unrecognized. Temozolomide is an essential medication for glioma [13]. Hence, for the first time, in the current study we analyzed the association of *TTC7B* with glioma.

## 2. Materials and Methods

### 2.1. Downloading and Preprocessing of Glioma Datasets

Clinical and transcriptome data of patients with glioma were downloaded from the TCGA (http://cancergenome.nih.gov/) and CGGA (http://www.cgga.org.cn/) database. From the CGGA database, the WHO grade, radiotherapy and chemotherapy status, 1p/19q codeletion, and *IDH* mutation status of 2,000 glioma samples were obtained [14]. In all, 325 specimens (dataset ID: mRNAseq_325) and 693 specimens (dataset ID: mRNAseq_693) of RNA-seq data comprised the 1,018 samples. The clinicopathological information and informed consent were obtained for all the samples. The work was authorized by the Institutional Review Board of Tiantan Hospital. From the TCGA database, 703 samples were downloaded, including 698 tumor samples and 5 paracarcinoma samples [15, 16]. After implementing data preprocessing in different datasets, a correlation analysis was conducted between the clinical variables and *TTC7B* expression.  Table 1 shows the comprehensive clinical data and the clinicopathological features of patients in the CGGA database. The R software (version 4.0.2) was utilized to carry out the gene expression and survival analyses. The Strawberry Perl software and the R software (version 4.0.2) enabled all the preprocessing procedures.

The article "TTC7B Is a Novel Prognostic-Related Biomarker in Glioma Correlating with Immune Infiltrates and Response to Oxidative Stress by Temozolomide" was retracted in 2023. Reasons: signs of a paper mill; suspected computer-generated content; unreliable results or conclusions; concerns about the data.

### 2.2. GEPIA Investigation of Survival and Expression

The Gene Expression Profiling Interactive Analysis (GEPIA) (http://gepia.cancer-pku.cn/index.html), an online repository, was employed to assess the link between *TTC7B* expression and survival of patients with glioma. The GEPIA website was used to examine the RNA sequence expression profile of 9,736 tumors and 8,587 normal specimens from the TCGA and GTEx studies. The GEPIA ‘survival' modules were used to evaluate the link between *TTC7B* expression and prognosis of patients with glioma. Furthermore, boxplots were used to depict the difference in *TTC7B* expression between the normal and tumor samples, with the disease conditions (normal or tumor) serving as variables.

### 2.3. Multivariate and Univariate Cox Model

Multivariate and univariate Cox analyses were conducted to evaluate the correlation of 1p/19q codeletion, treatment response, and overall survival (OS) with *TTC7B* expression. The survival program in R (version 4.0.2) was utilized to acquire the CGGA statistical analysis.

### 2.4. CIBERSORT Analysis

CIBERSORT is an extensively used algorithm for evaluating the cellular composition of intricate tissues according to their gene expression patterns because it produces findings that are consistent and predictable in majority of cancer cases. The LM22 signature-based algorithm was adopted upon data entry of the gene expression profiles exhibiting standard annotations to the CIBERSORT website application (http://cibersort.stanford.edu/). A further step was downloading the LM22, which is an annotated gene profile matrix representing the 22 distinct kinds of immune cells. This was accomplished via the use of the CIBERSORT online resource. CIBERSORT was employed to detect distinct kinds of immune cells, such as T cells, B cells, macrophages, natural killer cells, myeloid subsets, and dendritic cells, accurately and sensitively [17–20]. Data were classified based on the median *TTC7B* expression levels into high and low *TTC7B* expression groups to assess the differences in the proportion of immune cells between these groups.

The article "TTC7B Is a Novel Prognostic-Related Biomarker in Glioma Correlating with Immune Infiltrates and Response to Oxidative Stress by Temozolomide" was retracted in 2023. Reasons: signs of a paper mill; suspected computer-generated content; unreliable results or conclusions; concerns about the data.

### 2.5. TIMER Database Analysis

For the inclusive analysis of the TIICs, such as B cells, neutrophils, dendritic cells, CD4^+^ T cells, CD8^+^ T cells, and macrophages, the TIMER database (https://cistrome.shinyapps.io/timer/) was utilized by using the RNA-seq expression profile data [21, 22]. We used the “Gene” module plots to evaluate the link of *TTC7B* expression and immune infiltrate level with tumor purity.

### 2.6. Single-Cell Analysis

The Tabula Muris tool (https://tabula-muris.ds.czbiohub.org/) contains over 100,000 single-cell transcriptomes of 20 different tissues and organs. Through this database, we examined the associations between *TTC7B* expression levels and various types of cells and tissues, including endothelial cells and T lymphocytes. We also used fluorescence-activated cell sorting (FACS) to analyze the links between *TTC7B* expression and distinct types of cells.

### 2.7. Gene Set Enrichment Analysis

The Gene Set Enrichment Analysis (GSEA) (https://www.gsea-msigdb.org/) includes GO and KEGG pathway analysis, and was undertaken to examine the signaling pathways associated with *TTC7B* [23]. To evaluate the biological coherence and connections between each anticipated module, which was formed by correlating differently expressed mRNAs with distinct GO subsets, we performed GO analysis. An investigation of significant pathways linked to *TTC7B* expression was carried out using the KEGG analysis.

### 2.8. Quantitative RT-PCR

Total RNA was extracted from cell lines using the TRIzol reagent (Sigma-Aldrich, St. Louis, MO, USA). Then, 2 *μ*g RNA from each sample was subjected to quantitative reverse transcription-polymerase chain reaction using FastStart Universal SYBR ®Green Master (Roche, USA) on a Roche LightCycler 480 PCR System (Roche, USA). The cDNA was used as a template in a 20 *μ*l reaction volume (10 *μ*l of PCR mixture, 0.5 *μ*l of forward and reverse primers, 2 *μ*l of cDNA template, and an appropriate volume of water). PCR reactions were performed as follows: Cycling conditions started with an initial DNA denaturation step at 95°C for 30 s, followed by 45 cycles at 94°C for 15 s, at 56°C for 30 seconds, and at 72°C for 20 seconds. Each sample was examined in triplicate. Threshold cycle (CT) readings were collected and normalized to glyceraldehyde-3-phosphate dehydrogenase (*GAPDH*) levels in all samples using the 2^−ΔΔCT^ method. The mRNA expression levels of tumor tissues were compared with those of normal tissue controls. The sequences of primer pairs for the target genes are shown in Table 2.

The article "TTC7B Is a Novel Prognostic-Related Biomarker in Glioma Correlating with Immune Infiltrates and Response to Oxidative Stress by Temozolomide" was retracted in 2023. Reasons: signs of a paper mill; suspected computer-generated content; unreliable results or conclusions; concerns about the data.

### 2.9. Cell Culture and Drugs

Human glioma cell lines U-87 and U-251 were obtained from ATCC (Beijing Beina Chuanglian Biotechnology Institute), and cultured in F12 and DMEM medium containing 10% fetal bovine serum (Gibco, Carlsbad, CA, USA), respectively. Both cell lines were stored in a humidified incubator at 37°C with 5% CO_2_. Temozolomide was procured from MCE (USA, HY-17364), and dissolved in dimethyl sulfoxide (DMSO, Beyotime). Finally, it was cocultured with cells at a concentration of 20 *μ*M/ml.

### 2.10. Transwell Assay

Transwell assay was performed to assess the migration and invasion of glioma cells (U-87, U-251). Briefly, 5 × 10^4^ cells were inoculated into chambers coated (for invasion) or uncoated (for migration) with Matrigel (BD Biosciences, San Jose, CA). Serum-free medium was added to the upper layer and a complete DMEM medium was added to the lower layer. After 24 hours of incubation, migrating or invading cells were fixed with 4% paraformaldehyde, stained with 0.1% crystal violet, and counted under a light microscope.

## 3. Results

### 3.1. Relationship between *TTC7B* Expression and Glioma Survival Rates

*TTC7B* was found to be expressed at low levels in both, GBM [num (*T*) = 163 and num (*N*) = 207] and LGG [num (*T*) = 518 and num (*N*) = 207] (Figure 1(a)). Furthermore, low *TTC7B* expression was linked to an unfavorable OS [num (high) = 338 and num (low) = 338, *P* < 0.001; Figure 1(b)). A bipartite technique was utilized to classify the *TTC7B* expression levels in tumor and adjoining normal specimens into two groups, namely, high- and low-expression groups.

### 3.2. *TTC7B* Expression as an Independent Predictive Indicator for Individuals with Glioma

In univariate analysis, variables such as *TTC7B* expression (*P* < 0.001), PRS_type (*P* < 0.001), histology (*P* < 0.001), grade (*P* < 0.001), 1p19q_codeletion (*P* < 0.001), and *IDH*_mutation (*P* < 0.001) provide confirmation that *TTC7B* independently functions as a biological marker for patients with glioma (Figure 1(c)). Similarly,. In the multivariate model, factors linked to *TTC7B* expression (*P* = 0.005), notably, PRS_type (*P* < 0.001), *IDH*_codeletion (*P* < 0.001), 1p19q_codeletion (*P* < 0.001), and grade (*P* < 0.001), demonstrated that *TTC7B* independently served as a prognostic marker (Figure 1(d)). These findings demonstrate that *TTC7B* independently functions as a predictive marker for glioma and is highly correlated with several other variables associated with glioma. Moreover, the AUC of *TTC7B* expression was 0.57, 0.60, and 0.62 for 1-, 3-, and 5-year survival, respectively (Figure 1(e)). This illustrates that *TTC7B* has a satisfactory prognostic performance in anticipating the survival of patients with glioma.

The article "TTC7B Is a Novel Prognostic-Related Biomarker in Glioma Correlating with Immune Infiltrates and Response to Oxidative Stress by Temozolomide" was retracted in 2023. Reasons: signs of a paper mill; suspected computer-generated content; unreliable results or conclusions; concerns about the data.

### 3.3. The Association of *TTC7B* Expression with 1p/19q Codeletion and *IDH1* Phenotype Status in CGGA

The connection between *TTC7B* expression level and survival was evaluated in two separate datasets depending on the WHO grade and *IDH1* phenotype. The relationship between *TTC7B* expression pattern and WHO grade was examined and compared in two separate datasets (IDs: mRNAseq 693 and mRNAseq 325). Both datasets demonstrated a significant relationship between *TTC7B* expression pattern and WHO grade in gliomas (Figures 2(a) and 2(b)). These findings suggest that increased malignancy of glioblastoma was linked to attenuated *TTC7B* expression. Moreover, *TTC7B* expression was considerably downregulated in the *IDH* wild type group compared with the *IDH* mutant group, predicated on the two datasets characterized by *IDH* mutation status (Figures 3(a) and 3(b)) and computed using the ANOVA algorithm. *TTC7B* expression was remarkably reduced in the 1p/19q noncodeletion (noncodel) group (Figures 3(c) and 3(d)) when compared with the 1p/19q codeletion (*T*-test) group. These findings illustrate that *TTC7B* expression level was reduced in the I*DH* mutant and 1p19q codeletion groups.

### 3.4. *TTC7B* Overexpression Was Associated with a Favorable Chance of Survival in Primary Glioma

To examine the link between *TTC7B* expression and survival status (prognosis) in patients with WHO-graded glioma, a thorough survival analysis was conducted using the two CGGA datasets. *TTC7B* overexpression in dataset 1 (ID: mRNAseq_325) predicted favorable outcomes in primary glioma (*P* < 0.001; Figure 4(e)). Thus, we infer unequivocally that *TTC7B* overexpression level was correlated with better survival prognosis of patients with primary glioma.

### 3.5. Analysis of Multivariate Integrated Survival Data from the CGGA

To evaluate the therapeutic significance of *TTC7B*, factors such as chemotherapy (Figure 4(a)), radiation (Figure 4(b)), *IDH1* phenotypes (Figure 4(c)), and 1p/19q codeletion status (Figure 4(d)) were included in the multivariate analysis. In the 1p/19q-codeletion status group, lower *TTC7B* expression levels with 1p/19q codeletion predicted favorable survival outcomes compared with high *TTC7B* expression in patients without 1p/19q codeletion (Figure 4(d)). Additionally, *TTC7B* expression and chemotherapy were used to investigate the links between the survival probabilities. Elevated expression of *TTC7B* in the absence of chemotherapy was linked to favorable survival outcomes, whereas decreased expression of *TTC7B* in the presence of chemotherapy was associated with unfavorable survival results (Figure 4(a)). *TTC7B* seems to be substantially linked to all factors studied so far (*P* < 0.0001).

The article "TTC7B Is a Novel Prognostic-Related Biomarker in Glioma Correlating with Immune Infiltrates and Response to Oxidative Stress by Temozolomide" was retracted in 2023. Reasons: signs of a paper mill; suspected computer-generated content; unreliable results or conclusions; concerns about the data.

### 3.6. Association between TIICs and *TTC7B* Expression

We evaluated the correlation between TIICs of glioma and *TTC7B* expression level. Based on the CGGA specimens, the infiltration degree of immune cells, such as monocytes, activated mast cells, and T follicular helper cells, was considerably elevated in the high-expression group compared with the low-expression group. Further, based on the TCGA database, the infiltration degree of immune cells, such as plasma cells, T follicular helper cells, naïve B cells, and eosinophils, was considerably elevated in the high-expression group compared with the low-expression group. In addition, the CGGA (Figure 5(a)) and TCGA database (Figure 5(b)) revealed that NK cell activation (*P* < 0.001) was significantly reduced in the *TTC7B* high expression group.

### 3.7. *TTC7B* Expression Is Linked to the Degree of Immune Infiltration and OS in GBM and LGG Derived from TIMER

TIMER database was used to investigate whether the immune invasion level of glioma is related to *TTC7B* expression. In addition, we selected the *TTC7B* expression negatively linked to LGG purity. We identified a positive link between CD8^+^ T cell infiltration and *TTC7B* expression (*r* = 0.099, *p* = 3.03e − 02) (Figure 6(a)). In addition, the expression of *TTC7B* was intimately linked to the immunoinfiltrating microenvironment of macrophages, CD4^+^ T cells, and B cells in LGG. Furthermore, accumulation rates of GBM and LGG were found to be associated with DCs, macrophages, T cells neutrophils, and B cells (Figure 6(b)).

### 3.8. Investigation of *TTC7B* Expression and Cells from Various Organs by Single-Cell Analysis

We used the Tabula Muris database to study the relationship of *TTC7B* expression with cells. As demonstrated in Figure 7(a), brain tumors were linked to endothelial cells, basal cells, luminal epithelial cells of the mammary gland, stromal cells, and t-SNE of FACS cells. *TTC7B* was primarily linked to endothelial cells, basal cells, luminal epithelial cells of the mammary gland, and stromal cells, as illustrated in Figure 7(b).

### 3.9. Analysis of *TTC7B*-Related Pathways Using GSEA

We conducted GO and KEGG pathway analyses to probe into the probable bioactivities of *TTC7B*. We selected three pathways that were strongly linked with *TTC7B* expression and discovered that *TTC7B* is tightly linked to cellular metabolism and pathways. The KEGG pathway analysis illustrated that the MAPK, GnRH, and inositol phosphate metabolism signaling pathways exhibited a positive link to the elevated expression of *TTC7B*. In contrast, the three inversely linked categories were systemic lupus erythematosus, ECM receptor interaction, and cytokine-cytokine receptor interaction (Figure 7(c)). GO analysis revealed that *TTC7B* regulates response to oxidative stress (Figure 7(d)).

The article "TTC7B Is a Novel Prognostic-Related Biomarker in Glioma Correlating with Immune Infiltrates and Response to Oxidative Stress by Temozolomide" was retracted in 2023. Reasons: signs of a paper mill; suspected computer-generated content; unreliable results or conclusions; concerns about the data.

### 3.10. *TTC7B* Inhibits the Migration and Invasion of Glioma Cells

To assess the role of *TTC7B* in glioma progression, we examined *TTC7B* mRNA expression using qRT-PCR. PCR results indicated a decreased *TTC7B* expression in glioma patients. Transwell analysis (*in vitro*), including migration and invasion assays, revealed that migration and invasion capacity of glioma cells were reduced and *TTC7B* expression was increased with the use of temozolomide (Figure 8).

## 4. Discussion

Previous investigations have never identified the involvement of *TTC7B* gene in cancer. Hence, in the current study, we aimed to evaluate the role of *TTC7B* gene as prognostic biomarker of gliomas. We demonstrated that differences in the degree of *TTC7B* expression are linked to prognosis of patients with glioma. Additionally, *TTC7B* expression was found to independently serve as a prognostic marker for a positive prognosis. Moreover, the expression patterns of *TTC7B* were shown to be substantially correlated with a variety of clinical parameters, particularly pathological stage and tumor status. Furthermore, we found that *TTC7B* expression in glioma is linked to the expression of a variety of immune biomarkers and the degree of immune infiltration. Hence, the findings of the current investigation showed that *TTC7B* could have possible effects on tumor immunotherapy and might function as a promising cancer-related biological marker.

Using GEPIA, an online database, we discovered a link between *TTC7B* expression and prognosis of patients with glioma. The upregulated expression of *TTC7B* was shown to be linked to a positive prognosis. We obtained information from the TCGA database to better investigate the underlying processes and roles of *TTC7B* expression in cancers. *TTC7B* expression was shown to be associated with several clinical parameters, including pathological stage and tumor status, according to a statistical analysis conducted utilizing R-4.0.2. The results of multivariate analysis illustrated that *TTC7B* expression independently serves as a predictive factor for prognosis of patients with glioma. This research also compared the similarities between *IDH1* and *TTC7B* expressions. As indicated by WHO, *IDH1* phenotypes serve as a unique diagnostic technique for clinical usage and categorization of diffuse gliomas among adults is mostly determined by *IDH1* mutation status [3, 24, 25]. In this study, we investigated the differences between *IDH1* wild type and *IDH1*-R132 mutant groups. The elevated expression of *TTC7B* inhibits the progression of glioma to a malignant state, as evidenced by the reduced survival of the *IDH1*-R132 mutant group. Additionally, by comparing radiotherapy with chemotherapy, we were able to demonstrate the potential applications of *TTC7B*. Hence, the potential of *TTC7B* as a molecular predictor of prognosis of glioma was investigated in this research.

The article "TTC7B Is a Novel Prognostic-Related Biomarker in Glioma Correlating with Immune Infiltrates and Response to Oxidative Stress by Temozolomide" was retracted in 2023. Reasons: signs of a paper mill; suspected computer-generated content; unreliable results or conclusions; concerns about the data.

CIBERSORT analysis revealed a significant explicit link between *TTC7B* expression and NK cell infiltration levels in glioma. A similar pattern was seen in connections between gene biomarkers of various immune cells and *TTC7B* expression. This suggests that *TTC7B* has an important role in modulating the tumor immune microenvironment of glioma. Using the CIBERSORT algorithm we discovered that the proportion of NK cells was elevated in the high-expression group compared with the low-expression group. NK cells are viable immune effectors [26]. According to previous studies, NK cells may generate cytokines, including IFN-*γ* and TNF-*α*, which can suppress the progression, proliferation, and invasiveness of gliomas [27–32]. As a result, the favorable effects of *TTC7B* on glioblastoma are consistent with the role of high levels of NK cells, suggesting that *TTC7B* may have an impact on the OS of patients with glioma. Nevertheless, controlled experiments and multicenter clinical trials are required in the future to get a more precise understanding of the interaction between *TTC7B* and NK cells *in vivo*.

From GSEA analyses, the high-*TTC7B* expression group exhibited substantial enrichment of oxidative stress-related gene sets. In the previous research, in response to ionising radiation (IR) and chemotherapy, reactive oxygen species (ROS) are produced and are responsible for the mutagenic and cytotoxic effects of these agents. Increasing ROS levels cause DNA damage, lipid oxidation, and protein oxidation, ultimately leading to tumour cell death. Prior research identified putative pathways that might explain the association of *TTC7B* expression with better prognosis. Meanwhile, from qRT-PCR and Transwell analysis, *TTC7B* inhibits glioma cell migration and invasion, and temozolomide treatment increases TTC7B expression.

## 5. Conclusion

Overall, *TTC7B* serves as a predictive biological marker with prospective applications, and is associated with the immune infiltration and oxidative stress of gliomas. It might also function as a novel target for the regulation of immunosuppression. With the absence of a biological validation being performed, the study has several limitations. To elucidate its role in glioma, further clinical and experimental studies are required. However, it is expected that large sample sizes from CGGA and TCGA will help the subsequent investigation of gliomas.

The article "TTC7B Is a Novel Prognostic-Related Biomarker in Glioma Correlating with Immune Infiltrates and Response to Oxidative Stress by Temozolomide" was retracted in 2023. Reasons: signs of a paper mill; suspected computer-generated content; unreliable results or conclusions; concerns about the data.

## Figures and Tables

**Figure 1:** (a) Differential expression of *TTC7B* in GBM and LGG. (b) Survival curve analyzed by GEPIA in different *TTC7B* expression levels. (c, d) Multivariate and univariate Cox analysis of clinical-pathological factors and *TTC7B* expression. (e) The time-dependent receiver operating characteristic (ROC) curves of survival at 1-, 3-, and 5-years.

**Figure 2:** (a) Differences in *TTC7B* expression distribution in various WHO grades (dataset ID: mRNAseq_325). (b) Differences in *TTC7B* expression distribution in distinct WHO grades (dataset ID: mRNAseq_693).

**Figure 3:** The expression of *TTC7B* in CGGA dataset. (a) *IDH* status-stratified distribution (dataset ID: mRNAseq_325). (b) *IDH* status-stratified distribution (dataset ID: mRNAseq_693). (c) The 1p/19q-codeletion status distribution (dataset ID: mRANseq_325). (d) The 1p/19q-codeletion status distribution (dataset ID: mRNAseq_693).

**Figure 4:** Analysis of survival of CGGA patients in comparison to different *TTC7B* expression levels. (a) Chemotherapy, (b) radiotherapy, (c) IDH mutation, and (d) 1p/19q status. The Kaplan–Meier survival curve of *TTC7B* expression for GBM and LGG patients (e).

**Figure 5:** Proportion of 22 kinds of tumor-infiltrating immune cells in low- and high-*TTC7B* expression groups in tumor specimens. (a) CGGA dataset and (b) TCGA dataset.

**Figure 6:** (a) The *TTC7B* expression level is linked to the infiltrating levels of macrophages, T cells, and B cells in GBM and LGG. (b) OS is associated with the levels of DCs, neutrophils, B cells, macrophages, and T cells in GBM and LGG.

**Figure 7:** Single-cell analysis of *TTC7B* expression (a) Cells associated with brain tissue. (b) The proportion of *TTC7B* expressed in brain tissue. (c) KEGG analysis illustrated the pathways that were linked to *TTC7B*. (d) GO analysis illustrated the pathways that were linked to *TTC7B*.

**Figure 8:** *TTC7B* inhibits glioma cell migration and invasion, and temozolomide treatment increases *TTC7B* expression (a–d). Transwell assay images of migration and invasion in the NC and NECAP2 knockout groups, and quantitative analysis of migrating and invading glioma cells. (e) Results of quantitative analysis of TTC7B's mRNA expression in vivo. (f) Results of quantitative analysis of TTC7B's mRNA expression in U87 and U251 cell lines. (g) Results of quantitative analysis of RNF112 and NME5's mRNA expression in U87 cell lines. (h) Results of quantitative analysis of RNF112 and NME5's mRNA expression in U251 cell lines. ^∗^*p* ≤ 0.05, ^∗∗^*p* ≤ 0.01, ^∗∗∗^*p* ≤ 0.001 and ^∗∗∗∗^*p* ≤ 0.0001.

The article "TTC7B Is a Novel Prognostic-Related Biomarker in Glioma Correlating with Immune Infiltrates and Response to Oxidative Stress by Temozolomide" was retracted in 2023. Reasons: signs of a paper mill; suspected computer-generated content; unreliable results or conclusions; concerns about the data.

**Table 1:** Baseline of CGGA patients information.

	Total	Low-expression	High-expression	*χ* ^2^	*p*
PRS_type					
Primary	502	204	298	55.4292	0.0000
Recurrent	222	151	71		
Secondary	25	20	5		
Grade					
WHO II	218	45	173	186.0704	0.0000
WHO III	240	98	142		
WHO IV	291	232	59		
Gender					
Male	442	146	161	11.8564	0.0006
Female	307	229	213		
Age					
< = 41	342	139	203	2.4806	0.1553
>41	407	236	171		
Radio_status					
No	124	69	55	174.5180	<0.001
Yes	625	306	319		
Chemo_status					
No	229	94	135	51.2404	<0.001
Yes	520	281	239		
*IDH*_mutation_status					
Wildtype	366	274	92	0.4197	0.5171
Mutant	383	101	282		
1p19q_codeletion_status					
Noncodel	594	349	245	176.9779	<0.001
Codel	155	26	129		

**Table 2:** The sequences of primer pairs for the target genes.

Gene	Forward primer sequence (5′–3′)	Reverse primer sequence (5′–3′)
*TTC7B*	CCTGTCACCCACAGATCACC	CATGGACGGAGCCTGTCTCG
*RNF112*	CCTTTCCGGGAGAAAAGGCA	CCACGTGGACAAACATCTCC
*NME5*	TGGAGATATCAATGCCTCCACCT	CCAATCAGCTAGCCAAATCAAAGG
*GAPDH*	AATGGGCAGCCGTTAGGAAA	GCCCAATACGACCAAATCAGAG

## Data Availability

The data used in this article is downloaded from the public databases TCGA (http://cancergenome.nih.gov/) and CGGA (http://www.cgga.org.cn/). Readers can download and use it for free.
